# Clinical Application of Evoked Potentials in the Operation of Cervical Spondylotic Myelopathy with Different Imaging

This article has been retracted.

**DOI:** 10.1155/2022/4154278

**Published:** 2022-10-10

**Authors:** Xiaoli Ding, Zong Pan, Zongjun Ma, Zhaohui Ge

**Affiliations:** ^1^Department of Orthopedics, General Hospital of Ningxia Medical University, Yinchuan 750004, China; ^2^Department of Neurophysiology, General Hospital of Ningxia Medical University, Yinchuan 750004, China

## Abstract

**Objective:**

To observe the effects of improvement of cervical spondylotic myelopathy with different imaging signals after cortical somatosensory-evoked potentials on the functional recovery of postoperative patients and the effect of surgery.

**Methods:**

A total of 60 patients with cervical spondylotic myelopathy who were hospitalized in our hospital from January 2020 to December 2020 were selected and divided into a case group (30 cases) with MRI-indicated changes in intramedullary signals and a control group (30 cases) with MRI-indicated spinal cord changes. Intragroup and intergroup control studies were conducted through general observation indexes, neurological evaluation indexes, imaging, and evoked potential observation indexes. Somatosensory-evoked potentials were performed before operation, 1 week after operation, and 24 weeks after operation, and the JOA score of each patient was obtained before operation, 1 week after operation, and 24 weeks after operation.

**Results:**

The JOA score of 1 week after operation of the case group is (16.25 ± 1.54) and the control group is (11.89 ± 1.63), and there is a statistically significant difference (*P* < 0.05). The JOA score of the case group 24 weeks after operation is (25.27 ± 1.03) and the control group is (13.28 ± 1.03), and the difference is statistically significant (*P* < 0.05). The improvement rate of 1 week after operation and 24 weeks after operation was statistically significant between the two groups (*P* < 0.05). The case group improvement rate is (70.5 ± 8.72)% and the control group is (40.5 ± 9.81)%, and the difference is statistically significant between the two groups (*P* < 0.05).

**Conclusion:**

The preoperative intramedullary signal changes can be used as an effective index for patients with cervical spondylotic myelopathy to use somatosensory-evoked potentials to assess the prognosis of patients after surgery.

## 1. Introduction

Understanding the recovery of nerve function is the most urgent hope of spine surgeons. In the past clinical practice, clinicians mainly choose to arouse or conditioned reflex to judge the spinal cord injury and recovery level. In clinical practice, it is based on the physician's experience. The criteria for judging the level and the results of observation are not the same, and it is subjective. The imaging radiology technology developed in recent years has made up for the clinical judgment errors caused by the subjectivity of physicians to a certain extent. However, in recent years, somatosensory-evoked potential (SEP) is widely used by spine surgeons because of its high specificity to acute spinal cord and nerve injury. [1–3] Its application is easier, widely used, and simple and reliable results can be obtained, which is mainly used clinically in cervical spinal radiculopathy with compression of the spinal canal. The significant improvement of SEP waveform in most patients after spinal canal decompression can indicate that the compression is relieved and there is a good prognosis. This article focuses on surgery before and after SEP combined with imaging technology to improve cervical spondylotic myelopathy and its prognosis; relevant data analysis and research were carried out.

## 2. Materials and Methods

### 2.1. General Information

Sixty patients with cervical spondylotic myelopathy who were hospitalized in General Hospital of Ningxia Medical University from January 2020 to December 2020 were selected and divided into a case group and a control group. The case group was MRI-confirmed cervical spondylotic myelopathy (30 cases) with changes in intramedullary signal in which there were 16 males and 14 females aged 36-71 years, with an average of 47.5 years. The control group was MRI-confirmed cervical spondylotic myelopathy without changes in intramedullary signal (30 cases) in which there were 18 males and 12 females aged 33-65 years, with an average of 42.3 years.

### 2.2. Inclusion Criteria

The inclusion criteria are as follows: I. The imaging data of the cervical spine indicating the compression of the spinal cord and dural sac. II. The clinical symptoms were consistent with the imaging findings (instability of gait, stiffness of limbs, clumsy upper limbs, numbness, decreased muscle strength, muscle atrophy, and neck and shoulders pain). III. With or without upper extremity radiation pain. IV. All operations were performed by a senior physician, and the operation method was anterior cervical decompression and fusion.

### 2.3. Intraoperative-Evoked Potential Detection and Evaluation Criteria

The follow-up records were reviewed before the operation, 1 week after the operation, and 24 weeks after the operation. Each patient was scored systematically according to the Japanese Orthopedic Association (JOA), and each patient's record was recorded every time. Proceeding, calculated according to the formula of improvement rate (JOA postoperation-JOA preoperative)/(17-JOA preoperative) × 100%. Evaluate the curative effect of surgery based on 50% (improvement rate ≥50% was good, and <50 was generally). SEP monitoring was performed with the British SynerG10 evoked potential electromyography instrument before operation, 1 week after operation, and 24 weeks after operation. Place the disposable surface electrode on the patient's wrist to stimulate the median nerve of the upper limbs and the posterior part of the medial malleolus on both sides to stimulate the posterior tibial nerve of the lower limbs. The recording electrode was placed on the scalp C3 and C4 in which the stimulation frequency was 3.5 Hz, intensity was 25-35 mA, pulse width was 200 s, and average superimposition was 60-100 times (finger and toe micromovement shall prevail). [4, 5] Mainly observe the incubation period and amplitude of N19 and P22 waves and the changes of each waveform.

### 2.4. Efficacy Evaluation Criteria

The observation indexes were general observation indicators, neurological evaluation indicators, imaging, and evoked potential observation indicators, which were used to evaluate the effect of operation and the influence of related factors on the operation effect.

- General observation index: it records the patient's age, gender, occupation, smoking or not, whether there was a basic medical disease, the duration of the disease, the main symptoms and signs, whether there was a dysfunction in the urine and feces, whether there was intramedullary high signal on cervical MRI, the pain VAS score was followed up, and the VAS score of numbness was followed up before and after the operation.
- Neurological function evaluation indicator: the spinal cord injury function evaluation adopted the Japanese Orthopedic Association (JOA score) [6, 7]; the patient was evaluated before operation, 1 week after operation, and 24 weeks after operation; and JOA improvement rate was recorded.
- Imaging observation indicators: all cases were routinely performed cervical spine lateral X-rays, hyperextension and flexion X-rays, cervical CT and MRI before operation. Cervical anterior and lateral radiographs were performed within 1 week after surgery. Patients with intramedullary signal changes before surgery were followed up with MRI for 24 weeks.
- Evoked potential: recorded the changes of SEP potential before operation, 1 week after operation, and 24 weeks after operation and observed the change of evoked potential amplitude.

### 2.5. Statistical Analysis

The SPSS 20.0 software was used for statistical analysis, the measurement data was analyzed by using *t*-test, and the count data was analyzed by using chi-square test (*χ*^2^), and *P* < 0.05 was considered statistically different.

## 3. Results

### 3.1. Postoperative Patient Functional Recovery Results

The two groups of patients on the general observation indicators (age, gender, occupation, smoking or not, whether there were basic medical diseases, the duration of the disease, the main symptoms and signs, whether there was a dysfunction of urine and stool, whether there was intramedullary high signal on cervical MRI, the pain VAS score of followed up, and the VAS score of numbness of followed-up before and after the operation). There was no significant difference in the pain VAS score in the postoperative follow-up and the numbness in the preoperative and postoperative follow-up (*P* > 0.05).

The postoperative symptoms of all patients are improved compared with the preoperative symptoms. The changes in the JOA scores of the two groups in the postoperative follow-up are presented in Table 1. The data was statistically analyzed by Wilcoxon rank test, and the significance level was set at 0.05. The results showed that the preoperative comparison was compared with 1 week after operation and 24 weeks after operation. There was a significant difference in the increase of JOA score between the case group and the control group (*P* < 0.05).

### 3.2. Postoperative Surgical Results

In the case group and the control group, the improvement rate was calculated based on the JOA score of the patient 24 weeks after the operation. The statistical results are shown in Table 2 (the data results are statistically processed by Fisher's Test). The results showed that there were significant differences between the postoperative case group and the control group (*P* < 0.05). The postoperative improvement rate and average improvement rate of the case group were higher than those of the control group.

### 3.3. Comparison of MRI Results with Intramedullary Signal before and 24 Weeks after Operation

We compared the preoperative MRI results of patients with intramedullary signals with the MRI results of patients with intramedullary signals at 24 weeks after surgery; the intramedullary compression was significantly improved after the operation, as seen in Figure 1.

A is the preoperative cervical spine MRI examination result showing high signal in the spinal canal, B is the cervical spine MRI examination result 24 weeks postoperatively indicating that the compression is significantly improved compared with the preoperative compression, and the intramedullary signal has significant change.

### 3.4. Comparison of MRI Results before and 24 Weeks after Surgery without Intramedullary Signal

The preoperative MRI results of patients with no intramedullary signal were compared with the results of MRI at 24 weeks postoperatively in patients with no intramedullary signal, and there was a certain improvement compared with preoperative results, as seen in Figure 2.

A is the result of preoperative cervical spine MRI examination showing more low signals in the spinal canal, B is the result of cervical spine MRI examination 24 weeks after surgery indicating that the intramedullary low signal is reduced compared with preoperative examination, and the high signal is significantly increased.

### 3.5. Postoperative Follow-Up JOA Score Analysis

Comparison of the JOA Score of the case group at 1 week after operation (15.21 ± 1.34)%, 24 weeks after operation (18.22 ± 1.43)% with the case group before operation (7.53 ± 1.50)% were statistically significant (*P* < 0.05). It showed that the curative effect of the postoperative case group was significantly higher than that of the control group. Analysis of the improvement of the two groups was performed. It shows that the curative effect of the postoperative case group was significantly higher than that of the control group. The difference between the two groups was statistically significant (*P* < 0.05), and the difference between the two groups at 1 week and 24 weeks after the operation was statistically significant (*P* < 0.05). At the same time, the intragroup analysis of the case group was performed and the improvement rate was (70.5 ± 8.72)% and (40.5 ± 9.81) %, and the difference was statistically significant (*P* < 0.05). The statistical results are shown in Table 3.

## 4. Discussion

Cervical spondylotic myelopathy is one of the common clinical types of cervical spondylosis. Its pathological basis is the degeneration of facet joints and intervertebral discs, secondary to the formation of osteophytes in the backyard of adjacent vertebral joints that in turn leads to pairs of spinal cords or innervated spinal blood vessel compression, and patients may have various degrees of spinal cord dysfunction. [8–10] The current clinical practice is mainly surgery in order to improve blood supply to the spinal cord and reduce spinal cord lesions whose purpose is to relieve compression. In this study, both the case group and the control group have undergone spinal cord decompression, and the postoperative recovery satisfaction is excellent, indicating the clinical treatment effect of spinal cord decompression with the surgery is affirmative and stable and has a satisfactory curative effect. At present, more scholars are combining with spinal cord MRI examination technology on the basis of spinal cord decompression and believe that the morphological data analysis of the spinal cord before surgery can reduce the scope of spinal cord injury, but the postoperative recovery effect cannot be accurately evaluated. [11, 12] To a certain extent, it has affected the clinician's choice of treatment options for cervical spondylotic myelopathy. [13–16] In order to solve this problem, some scholars proposed to use somatosensory-evoked potential amplitude and latency to assess patients after spinal cord surgery to a certain extent recovery effect and changes in somatosensory-evoked potential amplitude and incubation period. [17–19] The main basis for evaluating the effect of surgical treatment is that the amplitude of the evoked potential can determine the number of neurons in response to the stimulus (when the number of neurons in response to the stimulus decreases, the amplitude curve of the evoked potential decreases) and then determine the electrical conductivity of the injured neurons to the evoked potential when the spinal cord is compressed [20–22], which indirectly reflects the number of spinal cord nerve injuries in the patients. The literature shows that the level of SEP amplitude combined with morphological testing can more accurately determine the patient's injury and recovery [23–25].

The change in amplitude during the operation can accurately judge the patient's later recovery, and a reduction of more than 50% indicates pathological damage. It is necessary to protect the spinal cord during the operation to avoid larger areas of damage. The latency period is to cooperate with amplitude that judges the degree of pathological damage. The latency period combined with the amplitude can more accurately judge the existence of pathological damage [26, 27]. Some scholars believe that a 50% reduction in volatility is too demanding for clinical requirements, and it is recommended to use higher than 60% as a warning value. Because of the lack of research results, this study did not adopt it.

The MRI manifestations of cervical spondylotic myelopathy mainly include the following: 1. The physiological curvature of the cervical spine becomes straight, and the physiological curvature disappears, which leads to instability of the vertebral body. The degeneration of the intervertebral disc protrudes posteriorly, MRI indicates that the signal is weakened, and the osteophyte shows a weakened signal pressure. 2. The morphological changes after the spinal cord is compressed and displaced which shows that the anterior and posterior edges of the cervical spinal cord are compressed in the sagittal position and is a bead-like change.The normal oval shape of the dural sac protruding forward or backward can be seen in the horizontal transverse position. The front and rear edges of the dural sac are flat, generally appearing as thin slices, concave inward. [28–31] Segment T2 is weighted as a high-signal or low-signal change and cervical spinal cord signals are involved [32–34].

The relationship between MRI imaging of cervical spondylotic myelopathy and patient prognosis has been generally recognized. It is generally believed that the increased T2 signal of the spinal cord indicates a poor prognosis. With the deepening of clinical and imaging technology cooperation and the study of many cases, many scholars have found that high signal does not necessarily indicate a poor prognosis. [17, 35–39] It is proposed that patients with high signal after surgery are better than those with low signal or no signal, and some scholars have found that whether there is high signal before surgery is not directly related to the degree of spinal cord compression or the efficacy of surgery. Some cases of hyperintensity can have reversible changes and have a good prognosis [40–42]. Some scholars have studied the changes of T1 and T2 that T1 low signal represents irreversible pathological damage, and there is a poor prognosis. It is considered that the signal level is high or low that can varying degrees predict the prognosis of cervical spondylosis to a certain extent [43–45]. In this study, the 30 cases in the case group are all hyperintensities, and the rank sum test was used for statistical processing. The comparability of the preoperative JOA scores of the two groups in this study did not affect the results of the study. The scores are similar in this study about the two groups of preoperative JOA that the case group is (8.23 ± 1.52) and the control group is (8.58 ± 1.24), and there is no difference in the preoperative JOA score (*P* > 0.05). In further studies, at 1 week after operation, JOA score of the case group is (16.25 ± 1.54) and the control group is (11.89 ± 1.63), and there is a statistically significant difference (*P* < 0.05). At 24 weeks after operation, JOA score of the case group is (25.27 ± 1.03) and the control group is (13.28 ± 1.03), and the difference is statistically significant (*P* < 0.05), and it is indicating that the curative effect of the postoperative case group is significantly higher than that of the control group. The results of the analysis of the relationship between postoperative intramedullary signal changes and improvement in the two groups of patients show that the preoperative case group and control group are (7.53 ± 1.50)% and (9.25 ± 1.72)% and that the difference between the groups is statistically significant (*P* < 0.05). The differences between the groups at 1 week after operation and 24 weeks after operation are statistically significant (*P* < 0.05). The case group analysis is performed, and the improvement rates are (70.5 ± 8.72)% and (40.5 ± 9.81)% and that the difference is statistically significant (*P* < 0.05). The author thinks through this research that the performance of cervical spondylotic myelopathy shown by MRI is a significant correlation with the clinical prognosis. We find by consulting the latest treatment guidelines of cervical spondylotic myelopathy that the surgical treatment of cervical spondylotic myelopathy should be carried out under the condition of evaluating the nerve function of SEP, and we should also monitor the recovery of nerve function after operation. The treatment effect can be significantly improved only by strictly following the instructions. For clinically suspecting cervical spondylotic myelopathy, cervical MRI should be routinely performed in order to cooperate with SEP to evaluate the patient's disease prognosis early and guide patients to carry out early rehabilitation exercises.

## Figures and Tables

**Figure 1:** MRI results before and 24 weeks after surgery with intramedullary signal.

**Figure 2:** MRI results before and after surgery without intramedullary signal.

**Table 1:** Comparison of changes in JOA scores between the two groups (mean ± *s*, score).

	Case group	Control group	*t*	*P-*value
Case number	30	30		
Preoperative	8.23 ± 1.52	8.58 ± 1.24	0.9773	>0.05
1 week after operation	16.25 ± 1.54	25.27 ± 1.03	10.65	<0.05
24 weeks after surgery	11.89 ± 1.63	13.28 ± 1.17	42.13	<0.05

**Table 2:** Analysis of the curative effect of postoperative cervical spondylotic radiculopathy (cases).

	*n*	Excellent	General	Distinguished achiever ratio	Average improvement rate (%)
				(%)	
Case group	30	28	2	93.3	55.21 ± 31.15
Control group	30	20	10	66.7	49.81 ± 15.88
*P* value		<0.05	<0.05	<0.05	<0.05

**Table 3:** Relationship between the changes of intramedullary signal and the improvement rate of the two groups of patients (*M* ± SD, %).

	Case group	Control group	T	*P-*value
Cases	30	30		
Preoperative	7.53 ± 1.50	9.25 ± 1.72	4.128	*P* < 0.05
1 week after operation	15.21 ± 1.34	10.22 ± 1.82	12.09	*P* < 0.05
24 week after operation	18.22 ± 1.43	12.31 ± 1.56	15.30	*P* < 0.05
Improvement rate %	72.5	42.3		

## Data Availability

The simulation experiment data used to support the findings of this study are available from the corresponding author upon request.

## References

[1] Yilmaz M., Yucesoy K., Erbayraktar R. S., Altinag R. S. (2021). Anterior hybrid construction of multilevel cervical disc disease and spondylotic spinal stenosis: surgical results and factors affecting adjacent segment problems. *Journal of Orthopaedic Surgery and Research*.

[2] Yu C. X., Li B., Xu Y. K. (2017). Altered functional connectivity of the periaqueductal gray in chronic neck and shoulder pain. *NeuroReport*.

[3] Yue X., Du Y. (2020). Altered intrinsic brain activity and regional cerebral blood flow in patients with chronic neck and shoulder pain. *Polish Journal of Radiology*.

[4] Abudouaini H., Wu T., Liu H. (2021). Partial uncinatectomy combined with anterior cervical discectomy and fusion for the treatment of one-level cervical radiculopathy: analysis of clinical efficacy and sagittal alignment. *BMC Musculoskeletal Disorders*.

[5] Ajiboye R. M., D’Oro A., Ashana A. O. (2017). Routine use of intraoperative neuromonitoring during ACDFs for the treatment of spondylotic myelopathy and radiculopathy is questionable: a review of 15, 395 cases. *Spine 1976*.

[6] Cao S., Zhao Y., Sun Y. (2021). Single-level cervical arthroplasty with prodisc-C vivo artificial disc: five-year follow-up results from one center. *Spine*.

[7] Chaiyamongkol W., Laohawiriyakamol T., Tangtrakulwanich B., Tanutit P., Bintachitt P., Siribumrungwong K. (2017). The significance of the trömner sign in cervical spondylotic myelopathy patient. *Clinical Spine Surgery: A Spine Publication*.

[8] Pilato F., Calandrelli R., Distefano M., Tamburrelli F. C. (2021). Multidimensional assessment of cervical spondylotic myelopathy patients. Usefulness of a comprehensive score system. *Neurological Sciences*.

[9] Chen G. L., Feng T. T., Xu S. T. (2018). [Clinical observation of percutaneous coblation nucleoplasty for the treatment of cervical spondylotic radiculopathy]. *Zhong Guo Gu Shang*.

[10] Cui Y., Zhou Y., Liu J., Duan D., Gong L., Li W. (2021). ACDF plus uncovertebrectomy versus ACDF alone for the treatment of cervical spondylotic radiculopathy: minimum 5-year follow-up. *Journal of Neurological Surgery Part A: Central European Neurosurgery*.

[11] Fujiwara Y., Izumi B., Fujiwara M. (2017). C2 spondylotic radiculopathy: the nerve root impingement mechanism investigated by para-sagittal CT/MRI, dynamic rotational CT, intraoperative microscopic findings, and treated by microscopic posterior foraminotomy. *European Spine Journal*.

[12] Goel A., Dharurkar P., Shah A., Gore S., Bakale N., Vaja T. (2019). Facetal fixation arthrodesis as treatment of cervical radiculopathy. *World Neurosurgery*.

[13] Zhang H. (2020). The value analysis of neuroelectrophysiological examination in the diagnosis of cervical spondylotic myelopathy. *Special Health*.

[14] Sakamoto T., Funaba M., Imajo Y. (2021). The impact of anterior spondylolisthesis and kyphotic alignment on dynamic changes in spinal cord compression and neurological status in cervical spondylotic myelopathy: a radiological analysis involving kinematic CT myelography and multimodal spinal cord evoked potentials. *Spine*.

[15] Guadarrama-Ortíz P., Choreño-Parra J. A., Carnalla-Cortés M., Sanchez-Garibay C., Palacios-Zuniga U. (2019). A case report of an intramedullary cervical teratoma in an adult patient with cervical spondylotic radiculopathy. *Neurocirugia*.

[16] Haijun M., Xiaobing Z., Bin G. (2020). Trans-interlamina percutaneous endoscopic cervical discectomy for symptomatic cervical spondylotic radiculopathy using the new Delta system. *Scientific Reports*.

[17] Taylor A. J., Combs K., Kay R. D., Bryman J., Tye E. Y., Rolfe K. (2021). Combined motor and sensory intraoperative neuromonitoring for cervical spondylotic myelopathy surgery causes confusion: a level-1 diagnostic study. *Spine*.

[18] Hirai S., Kato S., Nakajima K. (2021). Anatomical study of cervical intervertebral foramen in patients with cervical spondylotic radiculopathy. *Journal of Orthopaedic Science*.

[19] Huang Z., Tong Y., Fan Z., Zhao C., Gong P. (2020). Modified posterior percutaneous endoscopic cervical discectomy for the treatment of degenerative cervical spondylotic myelopathy caused by vertebral posterior osteophytosis. *World Neurosurgery*.

[20] Funaba M., Kanchiku T., Yoshida G. (2021). Efficacy of intraoperative neuromonitoring using transcranial motor-evoked potentials for degenerative cervical myelopathy: a prospective multicenter study by the monitoring committee of the Japanese society for spine surgery and related research. *Spine*.

[21] Jovicic M. D., Konstantinovic L. M., Grgurevic A. D. (2018). Validation of the neck disability index in Serbian patients with cervical radiculopathy. *Journal of Manipulative and Physiological Therapeutics*.

[22] Ke W., Zhi J., Hua W. (2020). Percutaneous posterior full-endoscopic cervical foraminotomy and discectomy: a finite element analysis and radiological assessment. *Computer Methods in Biomechanics and Biomedical Engineering*.

[23] Fustes O. H., Kay C. S. K., Lorenzoni P. J., Ducci R. D. P., Werneck L. C., Scola R. H. (2013). Somatosensory evoked potentials in Hirayama disease: a Brazilian study. *Surgical Neurology International*.

[24] Li C., Tang X., Chen S., Meng Y., Zhang W. (2019). Clinical application of large channel endoscopic decompression in posterior cervical spine disorders. *BMC Musculoskeletal Disorders*.

[25] Liang K. N., Feng P. Y., Feng X. R., Cheng H. (2019). Diffusion tensor imaging and fiber tractography reveal significant microstructural changes of cervical nerve roots in patients with cervical spondylotic radiculopathy. *World Neurosurgery*.

[26] Lin T., Wang Z., Chen G., Liu W. (2020). Predictive effect of cervical sagittal parameters on conservative treatment of single-segment cervical spondylotic radiculopathy. *World Neurosurgery*.

[27] Lin Z., Wang Z., Chen G., Lin T., Liu W. (2020). Is facet joint distraction associated with functional outcome in patients with cervical spondylotic radiculopathy treated with single-segment anterior cervical discectomy and fusion?. *World Neurosurgery*.

[28] Lu C. B., Ma Z. S., Hu J. B. (2020). Evaluation of anterior decompression surgical outcomes of proximal-type cervical spondylotic amyotrophy: a retrospective study. *Orthopaedic Surgery*.

[29] Ma J., Cheng Z., Jiang Z. (2019). Correlation analysis between C (7) slope and cervical sagittal parameters in short segment anterior cervical discectomy with fusion. *Zhongguo Xiu Fu Chong Jian Wai Ke Za Zhi*.

[30] McDonald M. A., Kirsch C. F. E., Amin B. Y. (2019). ACR appropriateness Criteria(®) cervical neck pain or cervical radiculopathy. *Journal of the American College of Radiology*.

[31] Mizouchi T., Katsumi K., Izumi T. (2020). Three-dimensional morphological analysis of cervical foraminal stenosis using dynamic flexion-extension computed tomography images. *Journal of Orthopaedic Science*.

[32] Shimohata K., Hasegawa K., Onodera O., Nishizawa M., Shimohata T. (2017). The clinical features, risk factors, and surgical treatment of cervicogenic headache in patients with cervical spine disorders requiring surgery. *Headache: The Journal of Head and Face Pain*.

[33] Wang Z., Rong Y., Tang P. (2021). Prevalence and predictive factors of asymptomatic spondylotic cervical spinal stenosis in patients with symptomatic lumbar spinal stenosis. *World Neurosurgery*.

[34] Wilkinson B. G., Chang J. T., Glass N. A., Igram C. M. (2021). Intraoperative spinal cord monitoring does not decrease new postoperative neurological deficits in patients with cervical radiculopathy or spondylotic myelopathy undergoing one or two level anterior cervical discectomy and fusion. *The Iowa Orthopaedic Journal*.

[35] Wilkinson B. G., Chang J. T., Glass N. A., Igram C. M. (2021). Intraoperative spinal cord monitoring does not decrease new postoperative neurological deficits in patients with cervical radiculopathy or spondylotic myelopathy undergoing one or two level anterior cervical discectomy and fusion. *The Iowa Orthopaedic Journal*.

[36] Nakanishi K., Tanaka N., Kamei N., Kotaka S., Ochi M., Adachi N. (2018). Evidence that impaired motor conduction in the bilateral ulnar and tibial nerves underlies cervical spondylotic amyotrophy in patients with unilateral deltoid muscle atrophy. *Spine Surg Relat Res*.

[37] Nakashima H., Kanemura T., Satake K. (2020). Reoperation for late neurological deterioration after laminoplasty in individuals with degenerative cervical myelopathy: comparison of cases of cervical spondylosis and ossification of the posterior longitudinal ligament. *Spine 1976*.

[38] Nwachuku E., Duehr J., Kulich S., Marker D., Moossy J. (2020). Cervical intramedullary spinal cavernoma in setting of unresolved myelopathy: a case report. *Surgical Neurology International*.

[39] Ramos M. R. D., Mendoza C. J. P., Yumol J. V., Joson R. S., Ver M. L. P., Ver M. R. (2021). Multilevel, percutaneous posterior cervical interfacet distraction and fusion for cervical spondylotic radiculopathy: clinical and radiographic outcomes. *Spine 1976*.

[40] Schulz C., Mauer U. M., Mathieu R. (2017). Clinical and radiological results after anterior cervical corpectomy with cage fusion - a retrospective comparison of PEEK vs. Titanium cages. *Zeitschrift für Orthopädie und Unfallchirurgie*.

[41] Shen W. S., Li C. F., Zhou Z. S., Zhai N. N., Pan L. P. (2020). MicroRNA-204 silencing relieves pain of cervical spondylotic radiculopathy by targeting GDNF. *Gene Therapy*.

[42] Sheng S. R., Wang K., Nisar M., Chen J. X., Wu A. M., Wang X. Y. (2018). A novel technique for cervical facet joint hyperplasia-spondylotic radiculopathy by laminar and lateral mass screw cofixations. *World Neurosurgery*.

[43] Ren J., Li R., Zhu K. (2019). Biomechanical comparison of percutaneous posterior endoscopic cervical discectomy and anterior cervical decompression and fusion on the treatment of cervical spondylotic radiculopathy. *Journal of Orthopaedic Surgery and Research*.

[44] Rho Y. J., Choe W. J. (2019). Double crush syndrome caused by cervical spondylosis and vertebral artery loop. *European Spine Journal*.

[45] Schell A., Rhee J. M., Holbrook J., Lenehan E., Park K. Y. (2017). Assessing foraminal stenosis in the cervical spine: a comparison of three-dimensional computed tomographic surface reconstruction to two-dimensional modalities. *Global Spine Journal*.

